The article "Silencing of Long Noncoding RNA HLA Complex P5 (HCP5) Suppresses Glioma Progression through the HCP5-miR-205-Vascular Endothelial Growth Factor A Feedback Loop" was retracted in 2024. Reasons: signs of a paper mill; suspected computer-generated content; unreliable results or conclusions; concerns about the data.

# Silencing of Long Noncoding RNA HLA Complex P5 (*HCP5*) Suppresses Glioma Progression through the *HCP5*-miR-205-Vascular Endothelial Growth Factor A Feedback Loop

**DOI:** 10.1155/2022/3092063

**Published:** 2022-06-20

**Authors:** Rui Cheng, Lei Ji, Haiyang Su, Lijun Wang, Ding Jia, Xiaohui Yao, Hongming Ji

**Affiliations:** Department of Neurosurgery, Shanxi Provincial People's Hospital, Taiyuan, 030012 Shanxi, China

## Abstract

Long noncoding RNA (lncRNA) HLA complex P5 (*HCP5*) is correlated with multiple diseases, especially cancers. However, it remains to be further studied whether *HCP5* is involved in the malignant behaviors of gliomas. This study is aimed at investigating the role and regulation mechanisms of *HCP5* in gliomas. *HCP5* expression in glioma tumor tissues and its association with glioma patients' survival were analyzed based on RNA-sequencing data. The expression of *HCP5* was also examined in glioma cells. Then, *HCP5* was downregulated in U251 cells and/or primary glioblastoma cells to explore its effects on cell proliferation and migration. The influence of *HCP5* downregulation on tumor growth was confirmed in xenograft mice. About the mechanism, we investigated whether *HCP5* functioned via interacting with microRNA- (miR-) 205 and regulating vascular endothelial growth factor A (*VEGF-A*) expression in gliomas. Results showed that *HCP5* upregulation was found in glioma tissues and cell lines. Patients with high *HCP5* expression showed lower survival probability and shorter survival time. *HCP5* downregulation inhibited cell proliferation and migration and mitigated tumor growth. miR-205 was downregulated in glioma cells. Knockdown of *HCP5* led to miR-205 upregulation and *VEGF-A* downregulation. miR-205 overexpression exhibited the similar effects as *HCP5* downregulation on cell viability and proliferation. And *VEGF-A* overexpression could reverse the effects of *HCP5* downregulation on cell viability and proliferation, as well as tumor growth. In conclusion, *HCP5* silencing suppressed glioma progression through the *HCP5*-miR-205-*VEGF-A* feedback loop.

## 1. Introduction

Gliomas are the type of primary neoplasias that occur in the brain, accounting for over eighty percent of primary brain tumors [1, 2]. Glioblastomas (GBMs), the most lethal primary gliomas, are grade IV gliomas classified by the World Health Organization [3, 4]. Currently, multiple therapeutic strategies have been applied in gliomas, such as surgical resection, chemotherapy, and radiotherapy; however, the prognosis is still very poor. The median survival is only 15 months in GBM patients, and 5-year survival rate postdiagnosis is proven to be 5.1% [5, 6]. Hence, the underlying mechanisms of glioma progression need further studies [4].

Long noncoding RNAs (lncRNAs), the transcripts exceeding 200 nucleotides in length, play important roles in cancers [7]. Increasing evidence reveals that many lncRNAs are dysregulated and implicated in the progression of many cancers, including gliomas, and they might act as therapeutic targets [8–13]. lncRNA HLA complex P5 (*HCP5*), firstly discovered in 1993, is correlated with a large majority of diseases, especially cancers [14]. *HCP5* was revealed to be a carcinogenic RNA contributing to the proliferation, migration, invasiveness, and angiogenic ability of follicular thyroid carcinoma cells [15]. *HCP5* promoted prostate cancer cell proliferation via interaction with microRNA- (miR-) 4656 [16]. Considering the reported malignant effects of *HCP5*, it is uncertain whether *HCP5* has a similar role in gliomas. Up to now, only one study reported that *HCP5* was upregulated in gliomas and its downregulation mitigated the malignant biological behavior of glioma cells [17].

miRs are endogenous short noncoding RNA strands with ~22 nucleotides that are responsible for 40%-60% of posttranscriptional regulation of gene expression [18]. Current thinking holds that lncRNAs function in cancers through serving as sponges for miRs. For example, *HCP5* contributed to the epithelial-mesenchymal transition (EMT) of colorectal cancer via interacting with miR-139-5p [19]. In anaplastic thyroid cancer, *HCP5* knockdown showed a tumor-suppressive function, which was proven to be correlated with the upregulation of miR-128-3p [20]. For gliomas, *HCP5* has been demonstrated to affect the malignant behavior of glioma cells via interacting with a tumor suppressor, miR-139, along with the alteration of Runt-related transcription factor 1 [17]. miR-205 is a highly conserved miRNA in many species. Studies have demonstrated that miR-205 could act as tumor promotor or suppressor in different cancers [21]. It has been demonstrated to be downregulated and functioned as a tumor suppressor in gliomas [22]. However, whether other miRs including miR-205 lie downstream of *HCP5* in gliomas still needs to be further studied.

This study is aimed at evaluating the role *HCP5* in gliomas both *in vitro* and *in vivo*. Moreover, the molecular mechanism of *HCP5* in the progression of gliomas was analyzed mainly focusing on the miR-205/vascular endothelial growth factor A (*VEGF-A*) axis.

## 2. Material and Methods

### 2.1. RNA-Sequencing Data Processing and Analysis

Based on the RNA-sequencing data (*n* = 9,736 for tumor samples; *n* = 8,587 for normal samples) from The Cancer Genome Atlas (TCGA) and Genotype-Tissue Expression (GTEx) projects, a web-based tool named Gene Expression Profiling Interactive Analysis (GEPIA: http://gepia.cancer-pku.cn/) was used to analyze gene expression [23]. The differential expression analyses of *HCP5* were performed via GEPIA in several cancer types, including cervical squamous cell carcinoma and endocervical adenocarcinoma (CESE; tumor: *n* = 306; normal: *n* = 13), cholangiocarcinoma (CHOL; tumor: *n* = 36; normal: *n* = 9), colon adenocarcinoma (COAD; tumor: *n* = 275; normal: *n* = 349), esophageal carcinoma (ESCA; tumor: *n* = 182; normal: *n* = 286), kidney chromophobe (KICH; tumor: *n* = 66; normal: *n* = 53), acute myeloid leukemia (LAML; tumor: *n* = 173; normal: *n* = 70), stomach adenocarcinoma (STAD; tumor: *n* = 408; normal: *n* = 211), and GBM (tumor: *n* = 163; normal: *n* = 207). Survival analysis of 224 glioma patients was also analyzed by GEPIA. These patients were assigned into two groups according to the median value of *HCP5* expression.

### 2.2. Cell Culture

Commercially available human GBM cell lines, including U87 MG (ATCC® HTB-14™) and A172 (ATCC® CRL-1620™), were purchased from the American Type Culture Collection (ATCC; Rockville, MD, USA). Normal human astrocytes (NHA) and human GBM cell line U251 were both obtained from the China Academia Sinica Cell Repository (Shanghai, China). GBM cells were cultured in Dulbecco's modified Eagle's medium (DMEM; Gibco, Carlsbad, CA, USA) containing 10% fetal bovine serum (FBS; Gibco), while NHA cells were grown in MCDB-131 medium (Sigma; St. Louis, MO, USA) containing 3% FBS and 10× G-5 Supplement (Gibco). Primary glioblastoma cell line was established as previously described [24]. Briefly, tumor tissue was obtained from one GBM patient. After removing the vessels, clotted blood, and charred tissue, sample was dissociated by Collagenase Type IVa (250 U/mL) and Pronase E (2.5 U/mL) for 1 h at 37°C. Then, cells were centrifuged at 300 × g for 5 min at 4°C, resuspended in DMEM containing 10% FBS, and put in a cell culture flask. The cell culture medium was changed every 2 days. Cells were all maintained in a humidified incubator with an atmosphere of 5% CO_2_ at 37°C.

### 2.3. Cell Transfection

Small interfering RNAs (siRNAs) against *HCP5* (si-HCP5#1, si-HCP5#2, and si-HCP5#3), their negative control (si-NC), miR-205 mimics, and scrambled miRs (NC mimics) were synthesized by GenePharma Co., Ltd. (Shanghai, China). Short hairpin RNA (shRNA) targeting *HCP5* (sh-HCP5) and its negative control (sh-NC) were cloned into pGPU6/GFP/Neo plasmid by GenePharma Co., Ltd. Full-length human *VEGF-A* gene was ligated into pcDNA3.1 plasmid (Invitrogen, Carlsbad, CA, USA), with empty pcDNA3.1 vector as a control (pcDNA3.1). These vectors were transfected into U251 cells using Lipofectamine 2000 (Invitrogen) following the manufacturer's instructions. Transfected cells were collected at 48 h after transfection to do the downstream experiments.

### 2.4. Cell Viability Assay

U251 or primary glioblastoma cells (2 × 10^3^ cells per well) were seeded in 96-well plates. After transfection, 20 *μ*L 3-(4,5-dimethylthiazol-2-yl)-5-(3-carboxymethoxyphenyl)-2-(4-sulfophenyl)-2H-tetrazolium (MTS) (Promega, Madison, WI, USA) per well was added on days 0, 1, 2, 3, 4, and 5, respectively. After 2 h incubation at 37°C, the absorbance value was measured by a plate reader at a test wavelength of 490 nm.

### 2.5. Scratch Wound-Healing Assay

U251 or primary glioblastoma cells (4 × 10^5^ cells per well) were seeded in 6-well culture plates. Cells were transfected with siRNA against *HCP5* (si-HCP5) or control siRNA (si-NC). 48 h after transfection, a linear scratch was created by a 200 *μ*L pipette tip, and cellular debris were removed by washing with phosphate buffer saline for three times. After culturing for another 48 h in serum-free medium, images of the scratched region were photographed by a microscope equipped with a camera (Nikon, Tokyo, Japan).

### 2.6. Proliferation Assay

Cell proliferative ability was determined by 5-ethynyl-2′-deoxyuridine (EdU) cell proliferation assay kit (RiboBio, Guangzhou, China) as previously described [25]. Firstly, transfected cells were seeded into 96-well plates. Following adhesion of the cells, 50 *μ*M EdU was added into each well, and cells were incubated at 37°C for 4 h, followed by fixation and permeabilization. Then, the cell nuclei were stained with 4,6-diamidino-2-phenylindole, dihydrochloride (DAPI). A fluorescence microscopy (Olympus, Tokyo, Japan) was employed to obtain the images. For each group, EdU-positive cells were counted as the average number in five random fields.

### 2.7. In Vivo Xenograft Experiments

Eight-week-old male C57BL/6 nude mice, obtained from the Guangdong Medical Laboratory Animal Center (Guangzhou, China), were divided into sh-HCP5 and sh-NC groups, or divided into pcDNA3.1-VEGF-A, pcDNA31, pcDNA31+sh-HCP5, and pcDNA3.1-VEGF-A+sh-HCP5 groups (*n* = 10 per group). After transfection with indicated plasmid, U251 cells (5 × 10^6^ cells per mouse) were subcutaneously injected into mice. Tumor volumes were recorded every 5 days from day 8 after injection according to the following formula: volume (mm^3^) = length × width^2^/2. All mice were euthanized by intraperitoneal injection of 100 mg/kg pentobarbital at 4 weeks postinjection, and tumor tissues were excised for further experiments. The animal experiments were carried out according to the Guide for the Care and Use of Experimental Animals of the National Institutes of Health, and the experimental protocol was approved by the Ethics Committee of the Shanxi Provincial People's Hospital (Shanxi, China).

### 2.8. Dual-Luciferase Reporter Assay

The binding sequence of miR-205 and *HCP5* was predicted by IntaRNA 2.0 online software (http:/http://rna.informatik.uni-freiburg.de/). The wild-type or mutant sequence of *HCP5* was cloned into pmirGLO dual-luciferase vector to construct luciferase reporter vectors, named HCP5 WT or HCP5 MT, respectively, and dual-luciferase reporter assay was carried out according to a previous study [26]. HEK293T cells were seeded into 96-well plates, followed by cotransfection with luciferase reporter vectors (HCP5 WT or HCP5 MT) and miRs (NC mimics or miR-205 mimics). After transfection for 48 h, the luciferase activity of transfected cells was determined by a Dual-Luciferase Reporter Assay System (Promega, Madison, WI, USA), as suggested by the manufacturer's instructions. Renilla luciferase was an internal reference.

### 2.9. Quantitative Reverse Transcription PCR (qRT-PCR)

Total RNA extracted by TRIzol reagent (Invitrogen) was used as a template for the synthesis of first-strand cDNA with the SuperScript® VILO™ cDNA Synthesis Kit (Invitrogen), and all steps were performed as the manufacturer's instructions. *HCP5* expression levels were obtained using a One Step SYBR® PrimeScript™ PLUS RT-RNA PCR Kit (TaKaRa Biotechnology, Dalian, China). The expression level of miR-205 was assessed using an All-in-One™ miRNA qRT-PCR reagent kit (GeneCopoeia Inc., Rockville, MD, USA). Besides, *VEGF-A* mRNA expression levels were measured by the PrimeScript™ 1st Strand cDNA Synthesis kit (TaKaRa) and the TB Green™ Premix Ex Taq™ II (TaKaRa) for reverse transcription and qRT-PCR, respectively. Primers used in this study are shown in Table 1, and the relative quantification of genes was calculated by the 2^-*ΔΔ*Ct^ method [16]. GAPDH was chosen as the housekeeping gene for *HCP5* and *VEGF-A*, whereas U6 was used as that for miR-205.

### 2.10. Western Blot Analysis

Proteins in U251 cells and tumor tissues were extracted using radioimmunoprecipitation assay (RIPA) lysis buffer containing 1 mM phenylmethanesulfonyl fluoride (PMSF) (both from Beyotime Biotechnology, Shanghai, China). After centrifugation, proteins in the supernatant were quantified using the BCA™ Protein Assay Kit (Pierce, Appleton, WI, USA). Then, extracted proteins were loaded (50 *μ*g/lane) and separated by dodecyl sulfate, sodium salt-polyacrylamide gel electrophoresis. Subsequently, proteins were transferred from the gel to the polyvinylidene difluoride membranes. Protein-bound transfer membranes were blocked by 5% nonfat milk for 1 h at room temperature, and then, membranes were successively incubated with respective primary antibodies (VEGF-A (ab214424) or GAPDH (ab181602), both were from Abcam (Cambridge, UK)) and HRP-conjugated secondary antibody (goat anti-rabbit, ab205718, Abcam, Cambridge, UK). Specific protein bands were visualized by using an ECL detection reagent (GE Healthcare, Braunschweig, Germany). Band intensity of VEGF-A was quantified using the ImageJ software (National Institutes of Health, Bethesda, MA, USA), with normalization to GAPDH.

### 2.11. Statistical Analysis

All experiments were repeated three times. Data are presented as the mean ± standard deviation (SD). Statistical analysis was carried out with GraphPad Prism 6 software (GraphPad, San Diego, CA, USA). The differences between two groups were analyzed by Student's *t* test. The differences among groups were compared by one-way analysis of variance (ANOVA) with Bonferroni post hoc test. Survival analysis was performed by the Kaplan-Meier method. *P* < 0.05 was considered as statistically significant.

## 3. Results

### 3.1. HCP5 Was Aberrantly Upregulated in Glioma Specimens and Commercial Glioma Cells

We firstly compared *HCP5* expression in cancer tissue samples and healthy control samples. Results in Figure 1(a) showed that *HCP5* levels in CESC, CHOL, COAD, ESCA, KICH, LAML, and STAD were all prominently higher than those in normal samples (all *P* < 0.05). Similarly, *HCP5* expression was significantly upregulated in GBM samples when compared to normal samples (*P* < 0.05, Figure 1(b)). Using the RNA-sequencing data from the Chinese Glioma Genome Atlas, the relationship between *HCP5* expression and the prognosis of 224 glioma patients was analyzed. Results revealed that patients with high *HCP5* expression had lower survival probability and shorter survival times than those with low *HCP5* expression (both *P* < 0.0001, Figure 1(c)). Moreover, the expression of *HCP5* in GBM cell lines (i.e., U87 MG, U251, and A172) was notably higher than that in normal NHA cells (all *P* < 0.05, Figure 1(d)). These results implied that *HCP5* overexpression might be correlated with GBM progression.

### 3.2. HCP5 Downregulation Inhibited Cell Proliferation and Migration and Mitigated Tumor Growth

The influences of *HCP5* on the malignant behaviors of GBM were analyzed via silencing *HCP5* both *in vitro* and *in vivo*. In this study, we designed three siRNAs against *HCP5*. *HCP5* levels in cells transfected with the three siRNAs against *HCP5* were significantly lower than those in cells with si-NC (*P* < 0.05, Figure 2(a)), and si-HCP5#2 and si-HCP5#3 showed higher knockdown efficiency than si-HCP5#1.  Figure 2(b) shows that cell viability was apparently mitigated after *HCP5* downregulation. Wound-healing assay in Figure 2(c) showed that knockdown of *HCP5* decreased cell migration, as the migration distance was obviously reduced following *HCP5* downregulation (*P* < 0.05). As depicted in Figure 2(d), compared with the si-NC group, the percentage of EdU-positive cells was decreased by *HCP5* downregulation (both *P* < 0.01). Furthermore, the effects of *HCP5* on GBM were investigated in nude mice. Tumor growth was slower in mice injected with *HCP5*-silenced U251 cells compared to those injected with U251 cells transfected with sh-NC (all *P* < 0.05, Figures 2(e) and 2(f)). Additionally, the effects of *HCP5* on GBM were also evaluated in primary glioblastoma cell line. We found that *HCP5* expression was higher in primary glioblastoma cells than in NHA cells (*P* < 0.05, Figure 2(g)). Downregulation of *HCP5* in primary glioblastoma cells significantly suppressed cell viability, migration, and the percentage of EdU-positive cells (all *P* < 0.05, Figures 2(h)–2(l)). These data suggested that *HCP5* was involved in tumorigenesis, as silencing of *HCP5* suppressed cell proliferation and migration *in vitro*, and repressed tumor growth *in vivo*.

### 3.3. HCP5 Downregulation Repressed Cell Proliferation via Interaction with miR-205

The regulatory mechanism of *HCP5* in GBM was further studied. miR-205 expression was found to be apparently downregulated in GBM cell lines including U87 MG, U251, and A172 cells relative to NHA cells (all *P* < 0.05, Figure 3(a)). We also found that miR-205 level was obviously higher in *HCP5*-silenced U251 cells than the si-NC group (*P* < 0.05, Figure 3(b)), which indicated that there might be a negative correlation between miR-205 and *HCP5* in GBM. The potential binding sites between *HCP5* and miR-205 were graphically marked in Figure 3(c). *HCP5* expression was prominently downregulated after miR-205 overexpression (*P* < 0.05, Figure 3(d)). Results in Figure 3(e) illustrated that the luciferase activity was markedly reduced in HEK293T cells that were cotransfected with HCP5 WT and miR-205 (*P* < 0.05), but a similar phenomenon was not found in cells with HCP5 MT. Moreover, both cell viability and the proportion of EdU-positive cells were dramatically lowered by miR-205 or si-HCP5. And compared with the si-HCP5 or miR-205 mimic group, cell viability and proliferation were further decreased in the si-HCP5+miR-205 mimic group (all *P* < 0.05, Figures 3(f) and 3(g)). These results confirmed that *HCP5* might act as a sponge of miR-205 in U251 cells.

### 3.4. HCP5 Downregulation Repressed GBM Proliferation through Downregulating VEGF-A

Finally, we investigated whether *HCP5* regulated GBM progression by modulating *VEGF-A* through miR-205. qRT-PCR assay showed that compared with the si-NC group, *VEGF-A* mRNA expression was significantly repressed in *HCP5*-silenced cells (*P* < 0.05, Figure 4(a)). Moreover, *HCP5* and *VEGF-A* mRNA levels were strikingly decreased while miR-205 expression was markedly increased in *HCP5*-silenced tumor tissues, compared to the sh-NC group (all *P* < 0.05, Figure 4(b)). Unsurprisingly, western blot results in Figure 4(c) indicated that VEGF-A protein expression levels were reduced both in *HCP5*-silenced U251 cells and tumor tissues. Additionally, a rescue experiment was used to further confirm whether *HCP5* functioned via regulating *VEGF-A*. Figure S1 illustrates that VEGF-A was successfully overexpressed in U251 cells transfected with pcDNA3.1-VEGF-A. In U251 cells, we found that *VEGF-A* overexpression not only increased cell viability and the proportion of EdU-positive cells but also reversed the influence of *HCP5* downregulation on these malignant behaviors (all *P* < 0.05, Figures 4(d) and 4(e)). Similarly, upregulation of *VEGF-A* promoted tumor growth and abrogated the effect of sh-HCP5 on tumor growth *in vivo* (all *P* < 0.05, Figures 4(f) and 4(g)). These data proved that *HCP5* downregulation functioned in GBM through downregulating *VEGF-A*.

## 4. Discussion

GBM is a devastating disease that is related to the dysregulation of multiple lncRNAs. In this study, we found that *HCP5* was aberrantly upregulated in GBM patients and cell lines. Patients with high *HCP5* expression showed shorter survival time. *In vitro* experiments proved that *HCP5* downregulation could suppress cell viability, migration, and proliferation in U251 cells. *HCP5* knockdown also repressed tumor growth in xenograft mice. Further experiments demonstrated that *HCP5* functioned via sponging miR-205 to positively regulate *VEGF-A* in gliomas.

Accumulating evidence has proven that *HCP5* was involved in the tumorigenesis of many cancers [27, 28]. Recently, researchers come to realize the importance of RNA sequencing in exploration for genetic mechanisms underlying human diseases [29]. RNA-sequencing data from TCGA and GTEx illustrated that *HCP5* was upregulated in many types of cancers including gliomas, which implied that *HCP5* possessed oncogenic potential in gliomas. In addition, lower survival probability and shorter survival time were shown in patients with high *HCP5* expression. *In vitro* experiments showed the increase of *HCP5* in GBM cells. The upregulation of *HCP5* in gliomas was consistent with a previous study [17]. Taken together, we hypothesized that *HCP5* might be an oncogenic gene in gliomas.

Two main distinguishing features of gliomas are rapid proliferation and angiogenesis [30]. Migration contributes to the high mortality of gliomas, and blocking cancer cell metastasis is considered to be a promising avenue for the treatment of this disease [31]. Studies have confirmed that *HCP5* promoted the proliferation and migration in clear cell renal cell carcinoma and gastric cancer [32, 33]. A previous study has pointed out that *HCP5* downregulation decreased cell viability and migration in U87 and U251 cells [17]. In line with these studies described above, this study found that *HCP5* knockdown inhibited the migration and proliferation of U251 and primary glioblastoma cells and prevented tumor growth in xenograft mice, which suggested that *HCP5* exerted a tumor-promotor role in gliomas.

Studying the molecular mechanisms of *HCP5* may provide innovative strategies for glioma therapy. The importance of miR-205 in gliomas has been evidenced in recent studies. For example, miR-205 was downregulated not only in glioma tissues but also in glioma cell lines, and it could inhibit EMT and tumor growth of gliomas [22]. miR-205 has been reported to be a target of many lncRNAs in gliomas [34, 35]. Hence, our study explored whether miR-205 was a target of *HCP5* in gliomas. We found that there was a negative correlation between miR-205 and *HCP5*, and *HCP5* could directly bind to miR-205 in GBM cells. Furthermore, miR-205 overexpression showed the similar effects as *HCP5* downregulation on GBM cell viability and proliferation. These results confirmed that *HCP5* functioned via targeting miR-205.

Many features of cancers such as migration, angiogenesis, and permeabilization of blood vessels are commonly correlated with *VEGF-A* [36]. Vascularization plays an important role in tumor progression, and aberrant angiogenesis is a hallmark of GBM [37]. Many studies indicated that there were binding sequences between miR-205 and *VEGF-A*, and miR-205 could target *VEGF-A* to inhibit the progression of multiple cancers [38–40]. Thus, we selected the *VEGF-A* as the downstream target gene of miR-205 and further analyzed whether *VEGF-A* was a downstream factor of *HCP5*. In this study, we found that *VEGF-A* was downregulated in *HCP5*-silenced U251 cells and tumor tissues. Moreover, the viability and proliferation of GBM cells as well as tumor growth could be enhanced by *VEGF-A* overexpression, and the upregulation of *VEGF-A* reversed the impacts of *HCP5* downregulation on these features. Our results, combined with previous studies, suggested that *HCP5* might affect glioma progression through the miR-205/*VEGF-A* axis.

## 5. Conclusions

Upregulation of *HCP5* was found in glioma tissues and cell lines. *HCP5* knockdown induced miR-205 upregulation, followed by the downregulation of *VEGF-A*, resulting in the repression of tumor cell proliferation and migration as well as tumor growth in gliomas. To our knowledge, this is the first time to report the correlation between *HCP5* and miR-205 in gliomas. Targeting *HCP5* and miR-205 might provide insight into a new strategy for glioma therapy.

## Figures and Tables

**Figure 1:** Potential correlation between *HCP5* overexpression and glioma. (a) The expression of *HCP5* in diverse cancer types, which was analyzed by GEPIA. (b) *HCP5* expression was assayed in GBM using GEPIA software. The boxes show the median and interquartile range, and the whiskers show the minimum and maximum values. (c) Prognostic value of *HCP5* in glioma patients detected by GEPIA. (d) The expression of *HCP5* in GMB cell lines and normal NHA cells, analyzed by qRT-PCR. Data are presented as the mean ± SD. ^∗^*P* < 0.05. TPM: transcripts per million.

**Figure 2:** *HCP5* downregulation inhibited cell viability and migration and mitigated tumor growth. U251 cells were transfected with si-NC, si-HCP5#1, si-HCP5#2, or si-HCP5#3. (a) *HCP5* expression was determined by qRT-PCR. (b) Cell viability was assessed by MTS assay. (c) Cell migration was examined by scratch wound-healing assay. (d) Proliferation was determined by EdU incorporation proliferation assay. U251 cells were transfected with sh-NC or sh-HCP5 and then injected into nude mice. (e) Tumors isolated from nude mice. (f) Tumor volume was recorded every 5 days from day 8 after injection. (g) *HCP5* expression in primary glioblastoma cells (pGCL) and NHA cells was measured by qRT-PCR. pGCL cells were transfected with si-HCP5#2. (h) *HCP5* expression level was analyzed. (i) Cell viability was assessed by MTS assay. (j, k) The migration of U251 cells was examined by scratch wound-healing assay after transfection with si-HCP5#2 and si-NC. And the wound-healing rate was measured. (l) EdU was used to examine the proliferation of pGCL cells. Data are presented as the mean ± SD. ^∗^*P* < 0.05; ^∗∗^*P* < 0.01.

**Figure 3:** *HCP5* downregulation repressed cell proliferation via interaction with miR-205. (a) miR-205 expression was assessed by qRT-PCR. U251 cells were transfected with si-NC or si-HCP5#2. Untransfected U251 cells acted as a control. (b) miR-205 expression was determined by qRT-PCR. (c) The binding sites between *HCP5* and miR-205 were predicted by IntaRNA 2.0. U251 cells were transfected with NC mimics or miR-205 mimics. Untransfected U251 cells acted as a control. (d) *HCP5* expression was assessed by qRT-PCR. (e) Relative luciferase activity was performed by dual-luciferase reporter assay. (f) Cell viability was evaluated by MTS assay in transfected U251 cells. (g) Proliferation was determined by EdU incorporation proliferation assay in transfected U251 cells. Data are presented as the mean ± SD. ^∗^*P* < 0.05; ^∗∗^*P* < 0.01.

**Figure 4:** Silencing of *HCP5* repressed GBM proliferation through downregulating VEGF-A. U251 cells were transfected with si-NC or si-HCP5#2. Untransfected U251 cells acted as a control. (a) *VEGF-A* mRNA expression was determined by qRT-PCR. U251 cells were transfected with sh-NC or sh-HCP5 and then injected into nude mice. (b) The expression levels of *HCP5*, miR-205, and *VEGF-A* mRNA in tumor tissues were examined by qRT-PCR. (c) VEGF-A protein levels in U251 cells and tumor tissues were determined by western blot analysis. (d) Cell viability was evaluated by MTS assay in transfected U251 cells. (e) Proliferation was detected by EdU incorporation proliferation assay in transfected U251 cells. U251 cells were transfected with pcDNA3.1-VEGF-A/pcDNA3.1 or cotransfected with sh-HCP5 and pcDNA3.1-VEGF-A/pcDNA3.1 and then injected into nude mice. (f) Tumors isolated from nude mice. (g) Tumor volume was recorded every 5 days from day 8 after injection. Data are presented as the mean ± SD. ^∗^*P* < 0.05.

**Table 1:** The primers used for real-time PCR.

Name	Primer sequences (5′ to 3′)
miR-205	Forward: GGGTCCTTCATTCCACCGG
	Reverse: CAGTGCGTGTCGTGGAGT
U6	Forward: GCTTCGGCAGCACATATACTAAAAT
	Reverse: CGCTTCACGAATTTGCGTGTCAT
HCP5	Forward: GACTCTCCTACTGGTGCTTGGT
	Reverse: CACTGCCTGGTGAGCCTGTT
VEGF-A	Forward: TCTTGGGTGCATTGGAGCCT
	Reverse: AGCTCATCTCTCCTATGTGC
GAPDH	Forward: CAATGACCCCTTCATTGACC
	Reverse: GACAAGCTTCCCGTTCTCAG

## Data Availability

The data used to support the findings of this study are included within the article.

## Abbreviations

lncRNA: Long noncoding RNA
HCP5: HLA complex P5
VEGF-A: Vascular endothelial growth factor A
GBM: Glioblastoma
miR: MicroRNA
EMT: Epithelial-mesenchymal transition
TCGA: The Cancer Genome Atlas
GTEx: Genotype-Tissue Expression
GEPIA: Gene Expression Profiling Interactive Analysis
CESE: Cervical squamous cell carcinoma and endocervical adenocarcinoma
CHOL: Cholangiocarcinoma
COAD: Colon adenocarcinoma
ESCA: Esophageal carcinoma
KICH: Kidney chromophobe
LAML: Acute myeloid leukemia
STAD: Stomach adenocarcinoma
ATCC: American Type Culture Collection
NHA: Normal human astrocytes
DMEM: Dulbecco's modified Eagle's medium
FBS: Fetal bovine serum
siRNAs: Small interfering RNAs
NC: Negative control
shRNA: Short hairpin RNA
MTS: 3-(4,5-Dimethylthiazol-2-yl)-5-(3-carboxymethoxyphenyl)-2-(4-sulfophenyl)-2H-tetrazolium
DAPI: 4,6-Diamidino-2-phenylindole, dihydrochloride
EdU: 5-Ethynyl-2′-deoxyuridine
qRT-PCR: Quantitative reverse transcription PCR
RIPA: Radioimmunoprecipitation assay
PMSF: Phenylmethanesulfonyl fluoride
SD: Standard deviation
ANOVA: One-way analysis of variance.

## Additional Points

*Highlights*. (i) *HCP5* was aberrantly upregulated in glioma samples and cells. (ii) *HCP5* silencing inhibited cell proliferation and migration and reduced tumor growth. (iii) *HCP5* downregulation repressed cell proliferation via interaction with miR-205. (iv) *HCP5* functioned via the miR-205/*VEGF-A* pathway.

## Supplementary Materials

Supplementary Materials Figure S1: VEGF-A was overexpressed in U251 cells transfected with pcDNA3.1-VEGF-A. U251 cells were transfected with pcDNA3.1 or pcDNA3.1-VEGF-A, and untransfected cells acted as a control. VEGF-A protein expression was determined by western blot analysis.
